This article has been retracted.

# Aus der Sektion Begutachtung der Deutschen Gesellschaft für Orthopädie und Unfallchirurgie in Zusammenarbeit mit der Deutschen Gesellschaft für Neurowissenschaftliche Begutachtung (DGNB): Bemessungsempfehlungen für muskuloskelettale Verletzungsfolgen in der Privaten Unfallversicherung

**DOI:** 10.1007/s00132-024-04499-2

**Published:** 2024-04-09

**Authors:** Marcus Schiltenwolf, Klaus Dresing, Johannes Eckert, Torsten Eyfferth, Peter Wolfgang Gaidzik, Martin Grotz, Sven Lundin, Klaus-Dieter Thomann, Bernhard Widder, Johannes Zeichen, DGOU Sektion Begutachtung

**Affiliations:** 1 Sektion Begutachtung, Deutsche Gesellschaft für Orthopädie und Unfallchirurgie, Berlin, Deutschland; 2 Konservative Orthopädie, Schmerzambulanz, Gutachtenambulanz, Klinik für Orthopädie, Universitätsklinikum Heidelberg, Schlierbacher Landstraße 200a, 69118 Heidelberg, Deutschland; 3 Klinik für Unfallchirurgie, Orthopädie und Plastische Chirurgie, Universitätsmedizin Göttingen, Göttingen, Deutschland; 4 Service- und Rehabilitationszentrum, BGU Berufsgenossenschaftliche Unfallklinik Frankfurt am Main, Frankfurt am Main, Deutschland; 5 Institut für Medizinrecht, Private Universität Witten/Herdecke gGmbH, Witten, Deutschland; 6 Geschäftsbereich Behandlungsfehler, Medizinischer Dienst Niedersachsen, Hannover, Deutschland; 7 BG-Klinikum Duisburg, Duisburg, Deutschland; 8 IVM – Institut für Versicherungsmedizin, Frankfurt, Deutschland; 9 Deutsche Gesellschaft für Neurowissenschaftliche Begutachtung (DGNB), Stuttgart, Deutschland; 10 Klinik für Unfallchirurgie und Orthopädie, Johannes Wesling Klinikum Minden, Minden, Deutschland

## Einleitung

In der PUV werden verbleibende Unfallfolgen nach muskuloskelettalen Verletzungen nach dem Prinzip der Invalidität bemessen. Bemessungstabellen haben eine lange Historie, die Thomann in dieser Zeitschrift bereits dargestellt hat [1]. Die Struktur der Bemessungstabellen hat eine lange Vorgeschichte. Wesentliche Elemente der aktuellen Einschätzungsempfehlungen gehen auf Schröter, Fitzek und Ludolph zurück [2–4].

Im folgenden Artikel werden die aktuell gültigen Tabellen der „Sektion Begutachtung“ der Deutschen Gesellschaft für Orthopädie und Unfallchirurgie dokumentiert. Dem orthopädisch-unfallchirurgischen Sachverständigen wird empfohlen, sich bei der Invaliditätsbemessung an den folgenden Tabellen zu orientieren. Die Tabellen entbinden den Gutachter nicht von seiner ärztlichen Verpflichtung, die Unfallfolgen umfassend, neutral und objektiv darzustellen und aus der Funktionsbeeinträchtigung den individuellen Invaliditätsgrad zu ermitteln.

Leistungspflicht für den Versicherungsträger besteht, wenn die körperliche oder geistige Leistungsfähigkeit dauerhaft beeinträchtigt ist (Invalidität). Die Invalidität durch Unfallfolgen wird gemäß „AUB 2020“ [5] nach der Gliedertaxe bemessen, sofern die betroffenen Körperteile oder Sinnesorgane dort genannt sind.

Für die Bemessung der Unfallfolgen in der PUV bestehen hierfür in der gängigen Gutachtenliteratur Tabellen [6–11], die rechtlich nicht bindend sind, jedoch Empfehlungscharakter haben. Die „Sektion Begutachtung“ der DGOU hat Unstimmigkeiten in diesen Tabellen erkannt und entwickelte eine aktualisierte Synopse der Bemessungsempfehlungen [12]. Hierbei erfolgten auch Modifikationen, soweit diese aus klinischer oder systematischer Sicht erforderlich erschienen. Ziel war es, bei jeder Bemessung die eindeutige Beschreibung der Funktionseinschränkungen zu prüfen. Die Sektion diskutierte alle einzelnen Bemessungen ausführlich, bis Einstimmigkeit erreicht werden konnte. Schließlich wurde dieser Diskussionsbeitrag der öffentlichen Diskussion angeboten (z. B. Jahrestagung der VSOU 2022 in Baden-Baden, DKOU 2022, Tagung zur privaten Unfallversicherung des Instituts für Versicherungsmedizin), woraus sich weitere Modifikationen ergaben. Zudem wurden Vorschläge ausführlich berücksichtigt und diskutiert, die eine Autorengruppe unter Leitung von Klemm et al. machte [13–16].

Ziel der aktuellen Bemessungstabellen ist eine Überwindung von Inkonsistenzen, die sich aus den bisher gängigen Tabellen ergaben. Weiterhin wurden Hinweise auf Operationspflichtigkeit gestrichen, da es sich um nicht duldungspflichtige Maßnahmen handelt. Damit bleiben solche Unfallfolgen ohne Konsequenz für die Bemessung. Verletzungsfolgen nach Wirbelbrüchen wurden auf die Bemessung der segmentbezogenen Funktionsstörung umgestellt. Bei den neurologischen Funktionsstörungen wurden die Leitsymptome der jeweiligen Ausfälle mit aufgelistet, um die Bemessung zu erleichtern.

## Bemessungsempfehlungen

Die Bemessung der Invalidität erfolgt einheitlich:

- Unfallfolgen der Extremitäten (und Sinnesorgane) werden in Zwanzigstel-Teilen des Gliederwerts des Verlusts bzw. des völligen Funktionsausfalls bemessen [17]. Nach der Rechtsprechung kann je nach Verletzungsbild sowohl der Ort der Verletzung als auch der Ort der Wirkung der unfallbedingten Schädigung die Zuordnung zur Gliedertaxe begründen [18].
- Unfallfolgen von Wirbelsäule, Becken, Thorax und Bauchdecken werden in Prozent Vollinvalidität bemessen.
- Unverändert seit 2009 bestimmt die vorrangige Unfallfolge die Invalidität. Nachrangige Befunde gehen ab einem Bemessungswert von mindestens 2/20 hälftig in der Gesamtbemessung subsummierend ein [4]. Eine Ausnahme stellen die Endoprothesenaufschläge dar, die voll berücksichtigt werden [4].

### Funktionsstörungen der Arm- und Beingelenke Vollversteifungen

(Tab. 1 und 2)

**Tab. 1:** Invalidität bei Vollversteifung der großen Gelenke an den Extremitäten in gebrauchsgünstiger Stellung (Tab. 2; [12])

Gelenk	Wert nach Gliedertaxe	Kommentar zur aktuellen Diskussion
Schulterhauptgelenk	^8/20^ A	Nicht mehr möglich sind: Beidhändiges Arbeiten an laufenden Maschinen. Mit der seitengleichen Hand: Tätigkeiten auf Schulterniveau und darüber, z. B. beidhändiges Ankleiden von Arbeitskleidung, Schutzbrillen. Tätigkeiten hinter dem Rumpf. Tätigkeiten seitengleich neben dem Rumpf mit Ziehen und Schieben. Beidarmiges sowie seitengleiches schweres Heben und Tragen, beidarmiges leichtes bis mittelschweres Heben und Tragen über Tischhöhe
Ellenbogengelenk (auch Unterarmdrehung)	^10/20^ A	Weiterhin soll die Versteifung des Ellenbogengelenks höher bemessen werden als die des Schultergelenks: Klemm et al. vergleichen Funktionsstörungen des versteiften Ellenbogengelenks mit dem auch im Schultergürtel versteiften Schultergelenk, berücksichtigt werden vorwiegend Aktivitäten, die Schulter- und Ellenbogenfunktionen zusammen erfordern [14]. Viele Aktivitäten sind bei versteiftem Ellenbogengelenk zusätzlich nicht möglich: Beidhändiges Arbeiten an laufenden Maschinen, mit Tastaturen. Heben von mittelschweren, schweren Lasten vom Boden. Beidarmiges Arbeiten am Boden und über Schulterhöhe. Mit der seitengleichen Hand zum Kopf für Anlegen von Schutzhauben, Arbeitsbrillen, Ankleiden des Oberkörpers, Halten eines Telefonhörers, Führen der Hand zum Mund für Essen, Trinken, Körperhygiene. Führen eines Lenkrads, Halten eines Fahrradlenkers. Durch die Versteifung der Unterarmdrehung sind zudem nicht möglich: Manuelle Tätigkeiten mit Anforderungen an schnelle Wechsel der Handhaltung der seitengleichen Hand z. B. an laufenden Maschinen, Blättern, Bedienen von Drehgriffen
Handgelenk	^6/20^ H	Weiterhin soll die Handgelenksversteifung mit 16,5 % des vollständigen Verlusts der Gebrauchsfähigkeit bemessen werden (entsprechend MdE 20 % im Bereich der GUV). Nicht möglich sind: Dauerhaftes Arbeiten mit betroffener Hand an Tastatur/Maus, Feinmotorische z. B. handwerkliche Tätigkeiten der betroffenen Hand
Hüftgelenk	^10/20^ B	Im Gegensatz zu historischen Bemessungsempfehlungen [19–21] stimmen wir Klemm et al. [14, 15] zu. Nicht möglich sind: Sitzen auf normalen Stühlen, Arbeiten mit gebücktem Oberkörper, Arbeiten im Knien, Hocken, Fersensitz oder Kriechen, Arbeiten auf Gerüsten oder Geländen mit Hindernissen, ein normales Fahrzeug führen, Fahrradfahren, dauerhaft Stehen ohne Möglichkeit von Steh- oder Gehpausen, alternierend Treppensteigen (nur mit Nachsetzen und erhöhtem Kraftaufwand)
Kniegelenk	^9/20^ B	Die Auswirkungen auf die Gebrauchsfähigkeit sind etwas geringer als beim versteiften Hüftgelenk. Nicht möglich sind: Sitzen mit gebeugtem Bein, in beengten Räumen (z. B. Toilette), Arbeiten im Knien, Hocken, Fersensitz oder Kriechen, Arbeiten auf Gerüsten oder Geländen mit Hindernissen (z. B. auf einem Schiff), ein normales Fahrzeug führen, Fahrradfahren
Oberes Sprunggelenk	^7/20^ F	Die Versteifung des oberen Sprunggelenks soll mit 14 % des vollständigen Verlusts der Gebrauchsfähigkeit bemessen werden (zum Vergleich: MdE 20 % im Bereich der Gesetzlichen UV). Nicht möglich sind: Arbeiten in der Hocke und im Knien, Arbeiten an schiefen Ebenen (z. B. Dachdecker), ein normales Fahrzeug führen, Gehen ohne Hinken
Unteres Sprunggelenk	^5/20^ F	5/20 Fußwert entsprechen 10 % der Gesamtinvalidität der versicherten Person (entsprechend der empfohlenen MdE im Bereich der Gesetzlichen UV). Nicht möglich sind: Aktivitäten auf unebenem Grund mit erhöhter Anforderung an die Balance
Oberes und unteres Sprunggelenk	^10/20^ F	Der halbe Fußwert ergibt sich aus der Subsumtion der Versteifungsbemessung von oberem und unterem Sprunggelenk. Nicht möglich sind: Arbeiten in der Hocke und im Knien, Arbeiten und Gehen an schiefen Ebenen (z. B. Dächer), ein normales Fahrzeug führen, Gehen ohne Hinken

*MdE* Minderung der Erwerbsfähigkeit, *GUV* Gesetzliche Unfallversicherung

**Tab. 2:** Gebrauchsgünstige Stellungen der Arm- und Beingelenke [6]. Versteifungen von Ellenbogen- und Handgelenk können auf Wunsch des Betroffenen abweichen

Gelenk	Gebrauchsgünstige Stellung
Schulter	In leichter Vorhalte (20–30°), Abspreizung 20–30°, Innendrehung 45° ± 10° und unwesentlicher Körperbreitenvermehrung
Ellenbogen	In knapper Rechtwinkelstellung mit 70–90° Beugung bei freier Unterarmdrehung
Unterarmdrehgelenk	Hand in leichter Einwärtsdrehung bis Mittelstellung (neutral bis 40° Pronation), Daumen nach oben bis innen-oben
Handgelenk	Leichte Streckung von 10–15° und nach ellenseitig um 0–10°
Daumensattelgelenk	Nach speichenseitig um 15–20°, zur Hohlhand um 30–40°, einwärtsgedreht um 10–15°
Fingermittel- und -endgelenke	Streckung bis leichte Beugung
Hüftgelenk	In leichter Beugung von 10–25°, Abspreizung 10–20°, Außendrehung 5–20°
Kniegelenk	In leichter Beugung von 5–10° und leichtem X von 5° und neutraler Drehung
Oberes Sprunggelenk	Leicht nach plantar, nach außen und valgisch jeweils um 10°
Unteres Sprunggelenk	Neutral
Großzehengrundgelenk	Gestreckt um 10–15°, zur zweiten Zehe um 5–10°

Mit dieser Empfehlung entfallen die Empfehlungen spezifischer Invaliditätswerte für Einstufungen in ungünstiger Stellung. In gebrauchsungünstiger Stellung erhöht sich die Bemessung um 1/20 bis 2/20 A/H/B/F-Wert. Bei einer Spitzfußstellung wird nach dem Beinwert bemessen.

### Schulterfunktionsstörungen mit Auswirkungen auf die Armfunktion

Die Bemessung orientiert sich an der Funktionsstörung in der Hauptbewegungsebene, dies ist die Arm-Vorhebung. In der Regel ist damit die vergleichbare Bewegungsstörung in der Seithebung miterfasst. Als Norm für die Abspreizung und Vorführung gilt ein Winkel von je 160–180°. Störungen der Rotation im Schultergelenk sind bei Störungen der Armhebung regelhaft zu erwarten und in der Bemessung enthalten (Tab. 3).

**Tab. 3:** Invalidität durch Bewegungsstörung im Schultergelenk, mit Auswirkungen auf die Armfunktion [12]

Funktionsstörung	Invalidität	Kommentar zur aktuellen Diskussion
Armhebung bis 120°	^2/20^ A	Von zusätzlicher Beeinträchtigung der Rotation ist auszugehen
Armhebung bis 90°	^4/20^ A	
Armhebung bis 60°	^6/20^ A	

### Schultergürtel und Schultergelenk mit Auswirkungen auf die Armfunktion

(Tab. 4)

**Tab. 4:** Invalidität durch Bewegungsstörung im Schultergelenk und Schultergürtel mit Auswirkungen auf die Armfunktion [12]

Funktionsstörung	Invalidität	Kommentar zur aktuellen Diskussion
*Schultergelenkdestruktion mit hochgradiger Bewegungsstörung, Abspreizen und Vorheben <* *30°, Außendrehung aufgehoben*	^10/20^ A	Das zerstörte Gelenk mit schmerzhafter Restbeweglichkeit ist funktionell schlechter als die schmerzfreie Versteifung, daher höhere Bemessung als von Klemm et al. [14] vorgeschlagen
*Instabilität des Schulterhauptgelenkes*		Abgestufte Bemessung nach Häufigkeit der Rezidivluxationen
Klinisch nachweisbar ohne Rezidivluxation	^1/20^ A	
Mit 1 Rezidivluxation	^2/20^ A	
Mit wiederholten Rezidivluxationen	^3/20^ A	
*Schultereckgelenksinstabilität*		Überstimmung zu sonstigen Empfehlungen [14]
Rockwood II + III	^1/20^ A	
Rockwood IV–V	^2/20^ A	
*Symptomatische Instabilität des Schlüsselbein-Brustbein-Gelenks*	^1/20^ A	
*Vollständiger Funktionsverlust der langen proximalen Bizepssehne*	^1/20^ A	

### Bewegungsstörungen des Ellenbogengelenks

Die Bemessung orientiert sich an der Funktionsstörung bei Streckung/Beugung und an der Unterarmdrehfähigkeit. Normal: Streckung/Beugung 10 – 0 – 140, Unterarmdrehung (Supination/Pronation) maximal 90 – 0 – 90 (Tab. 5).

**Tab. 5:** Invalidität durch Bewegungsstörungen des Ellenbogengelenks [8]

Funktionsstörung	Invalidität	Kommentar zur aktuellen Diskussion
*Streckung/Beugung 0° – 30° – 120°*		Die empfohlenen Werte sind historisch konstant, die Beeinträchtigung der Gebrauchsfähigkeit hat sich nicht verändert, um Absenkungen der Bemessung [14] zu begründen. Deutlich eingeschränkt sind: Tätigkeiten am Tastenbrett, Flaschenöffnen
Bei freier Unterarmdrehung	^3/20^ A	
Unterarmdrehung 45° – 0° – 45°	^5/20^ A	
*Streckung/Beugung 0° – 30° – 90°*		
Unterarmdrehung frei	^5/20^ A	
Unterarmdrehung 45° – 0° – 45°	^7/20^ A	
*Verlust der kompletten Unterarmdrehung bei freier Streckung und Beugung*	^6/20^ H*	Eine hälftige Absenkung der Bemessungsempfehlung [14] lässt die Bedeutung manueller Funktionen außer Betracht Nicht möglich sind: Manuelle Tätigkeiten mit Anforderungen an schnelle Wechsel der Handhaltung der seitengleichen Hand z. B. an laufenden Maschinen, Blättern, Bedienen von Drehgriffen
*Vollständiger Funktionsverlust der distalen Bizepssehne*	^2/20^ A	Überstimmung zu sonstigen Empfehlungen [14]

* Handwert, da die Handfunktion betroffen [12]

### Pseudarthrosen Ober- und Unterarm

Es gilt der Zustand bis zum Abschluss des 3. Jahres nach dem Unfall, unabhängig von (operativen) Sanierungsversuchen (Tab. 6).

**Tab. 6:** Invalidität durch Funktionsstörungen durch Pseudarthrosen des Ober- und Unterarms [12]

Funktionsstörung	Invalidität	Kommentar zur aktuellen Diskussion
*Oberarm-Pseudarthrose*		Keine sonstigen Empfehlungen
Straff und belastbar	^2/20^ A	
Instabil	^6/20^ A	
*Olekranon-Pseudarthrose*		
Straff und belastbar	^1/20^ A	
Mit Streckdefizit	^2/20^ A	
*Unterarm-Pseudarthrose*		
Straff und belastbar, Elle *oder *Speiche	^2/20^ A	
Straff und belastbar, Elle *und *Speiche	^4/20^ A	
Instabil Elle *oder *Speiche	^6/20^ A	
Instabil Elle *und *Speiche	^8/20^ A	

### Bewegungsstörungen im Handgelenk

Die Bemessung orientiert sich an der Funktionsstörung im Handgelenk und an der Unterarmdrehfähigkeit. Normal: Unterarmdrehung (Supination/Pronation) max. 90° – 0° – 90°, Dorsal‑/Volarflexion max. 60° – 0° – 60°, speichen-/ellenwärts max. 30° – 0° – 40° (Tab. 7).

**Tab. 7:** Invalidität durch Bewegungsstörungen des Handgelenks [22]

Funktionsstörung	Invalidität	Kommentar zur aktuellen Diskussion
*Bewegungseinschränkung Handgelenk konzentrisch zu ¼ bei*		–
Freier Unterarmdrehung	^2/20^ H	
*Bewegungseinschränkung Handgelenk konzentrisch zu ¼ bei*		
Eingeschränkter Unterarmdrehung 45° – 0° – 45°	^4/20^ H	
*Bewegungseinschränkung Handgelenk konzentrisch zu 1/2*		Eine konzentrische Bewegungseinschränkung um drei Viertel der Norm entspricht einer geringfügigen schmerzhaften Restfunktion mit geringerer Kraftentfaltung als bei Vollversteifung des Handgelenks und müsste daher höher bemessen werden als von Klemm et al. empfohlen [14]
Unterarmdrehung frei	^3/20^ H	
Bewegungseinschränkung Handgelenk konzentrisch zur Hälfte Unterarmdrehung 45° – 0° – 45°	^5/20^ H	

### Hand – Pseudarthrose, Nekrose

Die Mondbeinnekrose wurden als Entität gestrichen, sie ist äquivalent zwischen Kahnbeinpseudarthrose und karpalem Kollaps einzustufen. Das CRPS wurde herausgenommen, da die bisherigen Kriterien bei einem weiten Spektrum möglicher Funktionsstörungen zu ungenau erschienen, die Minderung der Gebrauchsfähigkeit nach CRPS soll individuell unter Bezug auf die Tabellenempfehlungen bemessen werden (Tab. 8).

**Tab. 8:** Funktionsstörungen durch Stabilitätsverlust der Handwurzel [12]

Funktionsstörung	Invalidität	Kommentar zur aktuellen Diskussion
*Kahnbeinpseudarthrose ohne Bewegungseinschränkung*		Keine sonstigen Empfehlungen
Straff und belastbar	^2/20^ H	
Instabil	^4/20^ H	
*Karpaler Kollaps*	^8/20^ H	

### Finger – Amputationsfolgen

(Tab. 9)

**Tab. 9:** Invalidität durch Fingerteilamputationen [12]

Funktionsstörung	Invalidität	Kommentar zur aktuellen Diskussion
*Teilverlust des Daumens*		Keine sonstigen Empfehlungen
Im Endgelenk	^12^/_20_ D	
Bis Mitte Grundglied	^16^/_20_ D	
*Verlust des Zeigefingers mit MH-Köpfchen (Adelmann)*	^4/20^ H	
*Verlust des Kleinfingers mit MH-Köpfchen*	^2/20^ H	
*Teilverlust der Finger II–V*		
Im Endgelenk	^8/20^ Fi	
Im Mittelgelenk	^14/20^ Fi	

Bei fehlender Belastbarkeit durch Neurombildung ^2^/_20_ Fi zusätzlich; *MH* Mittelhandknochen

### Versteifungen der Fingergelenke [10]

(Tab. 10)

**Tab. 10:** Invalidität durch Fingergelenkversteifungen [12]

Funktionsstörung	Invalidität	Kommentar zur aktuellen Diskussion
*Versteifung des Daumens*		Die Funktionsstörung des Daumens im Sattelgelenk ist nach dem Handwert zu bemessen. Die Versteifung ist i. A. durch Gelenkzerstörung begründet, wodurch die muskuloskelettalen Daumenfunktionen schmerzhaft verloren sind, was durch die empfohlene Bemessung bei Klemm et al. [14] nicht abgebildet wird
Im Sattelgelenk	^4/20^ H	
Im Grundgelenk	^4/20^ D	
Im Endgelenk	^4/20^ D	
Im Sattel- und Grundgelenk	^9/20^ H	
Im Grund- und Endgelenk	^8/20^ D	
*Versteifung der Finger II–V*		Versteifungen der Grundgelenke sollen höher, der Mittelgelenke niedriger bemessen werden in Übereinstimmung mit Klemm et al. [14]
Im Grundgelenk	^8/20^ Fi	
Im Mittelgelenk	^6/20^ Fi	
Im Endgelenk	^4/20^ Fi	
Im Grund- und Mittelgelenk	^14/20^ Fi	
Im Mittel- und Endgelenk	^10/20^ Fi	

### Fingersehnen, -bänder

(Tab. 11)

**Tab. 11:** Invalidität durch Funktionsstörungen der Fingersehnen und Instabilität [12]

Funktionsstörung	Invalidität	Kommentar zur aktuellen Diskussion
Streckdefizit von mehr als 10° am DIP nach Strecksehnenabriss	^2/20^ Fi	In Übereinstimmung mit Klemm et al. [14]
Ulnare Seitenbandinstabilität am Daumengrundgelenk	^2–4/20^ D	Abgestufte Bemessung ja nach Ausprägung der Instabilität [14]

*DIP* distales Interphalangealgelenk

### Sensibilitätsstörungen der Finger durch Nervenschäden

(Tab. 12)

**Tab. 12:** Invalidität durch Sensibilitätsstörungen der Finger [11]

Funktionsstörung	Invalidität	Kommentar zur aktuellen Diskussion
**Am Daumen**		Keine sonstigen Empfehlungen
*Nur Daumenbeere*		
Volar: nur speichenseitig	^4/20^ D	
Volar: nur ellenseitig	^4/20^ D	
Volar: ellen- und speichenseitig	^8/20^ D	
**An den Fingern II–V**		Keine sonstigen Empfehlungen
*Nur Fingerbeere*	^4/20^ Zf/Fi	
Volar – einseitig	^8/20^ Zf/Fi	
Volar – beidseitig	^10/20^ D/Zf/Fi	
Gesamter Finger	^12/20^ D/Zf//Fi	

Betrifft die Sensibilitätsstörung nicht nur die Fingerbeere, sondern den ganzen Finger werden ^1^/_10_ D/Zf/Fi zusätzlich gewertet

### Bewegungsstörung des Hüftgelenks

Die Bemessung orientiert sich an der Funktionsstörung in der Hauptbewegungsebene. Normal: Streckung/Beugung 10° – 0° – 130° (Tab. 13).

**Tab. 13:** Invalidität durch Bewegungsstörungen des Hüftgelenks [12]

Funktionsstörung	Invalidität	Kommentar zur aktuellen Diskussion
Streckung/Beugung 0° – 0° – 90°	^2/20^ B	Übereinstimmung mit Klemm et al. [15]
Streckung/Beugung 0° – 0° – 60°	^4/20^ B	
Streckung/Beugung 0° – 0° – 30°	^6/20^ B	
*Zusätzliches Streckdefizit bzw. Abduktions‑/Adduktions‑/Rotationskontrakturen*		–
10–20°	Erhöhung um ^1/20^ B	
30° (und mehr)	Erhöhung um ^2/20^ B	

### Endoprothesen

Für Minderbelastbarkeit/Lockerungsgefahr und zu erwartendem Prothesenwechsel wird abhängig vom Lebensalter ein Zuschlag gegeben. Bei Schulter‑, Ellenbogen- und Sprunggelenkendoprothesen sind jeweils um ^1^/_20_ höhere Zuschläge begründet (Tab. 14).

**Tab. 14:** Invalidität durch Minderbelastbarkeit/Lockerungsgefahr und zu erwartendem Prothesenwechsel [12]

*Basisbewertung* nach Funktion, zuzüglich Zuschlag nach Lebensalter, *Bemessung des Zuschlages:*		
Lebensalter (Jahre)	Zuschlag	Kommentar zur aktuellen Diskussion
15–20	11/20	Im Gegensatz zur Einschätzung von Klemm et al. [13] ist mit zunehmender Standzeit der Endoprothese mit Wechseloperationen, Verlust an Knochenmasse zur Verankerung und Gebrauchsfähigkeit, letztlich mit Verlust der Gelenkgebrauchsfähigkeit zu rechnen [23, 24], die Ausfallwahrscheinlichkeit einer Endoprothese ist bei posttraumatischen Arthrosen zudem höher, die bei jüngeren Betroffenen häufiger auftreten [25], auch wenn der Anteil junger und sehr junger Betroffener mit posttraumatischer Arthrose gering ist.
21–25	10/20	
26–30	9/20	
31–35	8/20	
36–40	7/20	
41–45	6/20	
46–50	5/20	
51–55	4/20	
56–60	3/20	
61–65	2/20	
66 und mehr	1/20	

### Hüftkopf

Auf die Angabe „kleines Kopfareal“ wurde verzichtet, da dies unpräzise und nicht messbar ist, stattdessen wird der Befund Nekrose ohne Progredienz eingeführt. Die Prothesenpflichtigkeit wurde gestrichen, da es sich um eine nicht duldungspflichtige operative Maßnahme handelt (Tab. 15).

**Tab. 15:** Invalidität durch Funktionsstörung durch Strukturstörungen des Hüftgelenks [12]

Funktionsstörung	Invalidität	Kommentar zur aktuellen Diskussion
*Hüftgelenkverlust (Girdlestone)*	^14/20^ B	Keine sonstigen Vorschläge
*Hüftkopfnekrose*		
Nekrose ohne Progredienz, geringe Funktionsstörung	^4/20^ B	
Nekrose mit Progredienz je nach Funktionsstatus	Individuelle Bemessung	

### Bewegungsstörungen im Kniegelenk

Die Bemessung orientiert sich an der Funktionsstörung bei Streckung und Beugung. Normal: 5° – 0° – 135° (Tab. 16).

**Tab. 16:** Invalidität durch Bewegungsstörungen des Kniegelenks [12]

Funktionsstörung	Invalidität	Kommentar zur aktuellen Diskussion
Beugung bis 90°	^2/20^ B	Die Beugung bis 90° beeinträchtigt den alternierenden Treppengang, das Radfahren, das Arbeiten im Knien, Hocken, Fersensitz oder Kriechen, in beengten Räumen. Die vorgeschlagene Halbierung der Bemessung ist daher nicht angemessen für diese Gebrauchsminderung
Beugung bis 60°	^4/20^ B	
Beugung bis 30°	^6/20^ B	
*Zusätzliches Streckdefizit*		Keine sonstigen Vorschläge
Bis 10°	Erhöhung um ^1^/_20_ B	
Bis 20°	Erhöhung um ^5/20^ B	
Über 20°	Erhöhung um ^7/20^ B	

### Instabilitäten des Kniegelenks

Die Bemessung orientiert sich am Ausmaß der Instabilität und ihrer Kompensierbarkeit.

Analog ist diese Bemessung auch auf andere Gelenke übertragbar. Die Erhöhung bei ungenügender/fehlender muskulärer Kompensation wurde hier gestrichen, da bei Muskelminderung bereits erfasst. Bei der Bemessung ist zu beachten, dass bei Instabilität plus Indikatoren auf Arthroserisiko (Kreuzbandverletzung und Meniskusverlust) die Arthroserate ansteigt und in der Bemessung berücksichtigt werden sollte, z. B. zusätzlich 1/20 B (Tab. 17 und 18).

**Tab. 17:** Invalidität durch Instabilitäten des Kniegelenkes [12]

Instabilität	Invalidität	Kommentar zur aktuellen Diskussion
Leichtgradig (+ nur ein Band)	^1^/_20_ B	In Übereinstimmung mit Klemm et al. [15]
Leichtgradig (+ kombiniert)	^3/20^ B	
Mittelgradig (++ nur ein Band)	^3/20^ B	
Mittelgradig (++ kombiniert)	^6/20^ B	
Hochgradig (+++ nur ein Band)	^5/20^ B	
Hochgradig (+++ kombiniert)	^10/20^ B

**Tab. 18:** Bewertungsschema nach Ausmaß der Instabilität/Bandnachgiebigkeit [12]

Kategorie	Aufklappbarkeit/Vor‑/Rückschub
0	= 0–2 mm
(+)	= grenzwertiger Befund
+	= 3–5 mm
++	= 6–10 mm
+++	= > 10 mm

### Bewegungsstörung des oberen Sprunggelenks nach *Fußwert*

Die Bemessung orientiert sich primär an der Funktionsstörung beim Heben/Senken des Fußes im oberen Sprunggelenk. Normal: Heben/Senken 20^°^ – 0° – 40° (Tab. 19).

**Tab. 19:** Invalidität durch Bewegungsstörungen im oberen Sprunggelenk [12]

Funktionsstörung	Invalidität	Kommentar zur aktuellen Diskussion
10° – 0° – 30°	^3/20^ F	Vorgeschlagen werden Verringerungen der Bemessung zwischen 40 und 66 % [15]. Dies ist der Gebrauchsbeeinträchtigung beim Abrollvorgang, Gehen auf geneigtem Grund nicht angemessen
0° – 0° – 30°	^6/20^ F	
0° – 0° – 20°	^7/20^ F*	
*Bei zusätzlichem Bewegungsdefizit im unteren Sprunggelenk (USG)*		
Gering	Kein Zuschlag	Keine Änderungsvorschläge [15]
^1^/_3_	Erhöhung um ^2/20^ F	
^2^/_3_	Erhöhung um ^3/20^ F	

* Funktionell vergleichbare Situation wie Vollversteifung des oberen Sprunggelenkes in gebrauchsgünstiger Stellung, deshalb gleiche Bemessung

#### Bewegungsstörung des oberen Sprunggelenks nach *Beinwert*

Normal: Heben/Senken des Fußes 20° – 0° – 40°. Die Bemessung orientiert sich am Ausmaß des Spitzfußes (Tab. 20).

**Tab. 20:** Invalidität durch Bewegungsstörungen des oberen Sprunggelenks mit Auswirkungen auf das Kniegelenk [12]

Funktionsstörung	Invalidität	Kommentar zur aktuellen Diskussion
OSG 0 – 10 – 30	^5/20^ B	Diese Funktionsstörungen wirken sich auf das Kniegelenk aus, daher Bemessung nach dem Beinwert im Gegensatz zu Klemm et al. [15]
OSG 0 – 20 – 30	^6/20^ B	
OSG 0 – 30 – 30	^7/20^ B	
*Bei zusätzlichem Bewegungsdefizit im unteren Sprunggelenk (USG):*		
Gering	Kein Zuschlag	Keine sonstigen Vorschläge
^1^/_3_	Erhöhung um ^2^/_35_* B (= ^2/20^ F)	
^2^/_3_	Erhöhung um ^3^/_35_* B (= ^3/20^ F)	

*OSG* oberes Sprunggelenk

* Abweichung von der Systematik mit ^1^/_20_-Raster zwecks identischer Bemessung nach Bein- und Fußwert abgestellt auf die Musterbedingungen. Bei individueller Vertragsgestaltung (z. B. Beinwert = 80 % der Versicherungssumme) erfolgt die Zuschlagsbemessung analog (z. B. mit ^2^/_40_ bzw. ^3^/_40_ Beinwert)

### Fuß- und Zehenverluste

(Tab. 21)

**Tab. 21:** Invalidität durch Fuß- und Zehenverluste [12]

Funktionsstörung	Invalidität	Kommentar zur aktuellen Diskussion
Amputation in Höhe der Chopart-Gelenklinie	^12/20^ F	Keine sonstigen Vorschläge
Amputation in Höhe der Lisfranc-Gelenklinie	^10/20^ F	
Verlust im Mittelfußbereich (Sharp)	^8/20^ F	
Großzehe mit Mittelfußknochen	^4/20^ F	

### Groß- und Kleinzehenversteifungen

Ist die Abrollfähigkeit des ganzen Fußes beeinträchtigt, wird nach dem Fußwert bemessen (Tab. 22).

**Tab. 22:** Invalidität durch Versteifungen von Zehengelenken [12]

Funktionsstörung	Invalidität	Kommentar zur aktuellen Diskussion
*Großzehe*		Die Beugestellung der Großzehe beeinträchtigt den Abrollvorgang des Fußes. Daher Bemessung nach dem Fußwert im Gegensatz zum Vorschlag von Klemm et al. [15]. Dagegen ist die Grundgelenkversteifung in Überstreckstellung funktionell günstig und soll daher nicht mit 6/10 Gz [15] bemessen werden
Grundgelenkversteifung in Beugestellung	^3/20^ F	
Grundgelenkversteifung in Neutralstellung	^2/20^ F	
Grundgelenkversteifung in Überstreckstellung	^8/20^ Gz	
Endgelenkversteifung in Streckstellung	^8/20^ Gz	
*Kleinzehen (II–V, alle Gelenke)*		Keine Änderungsvorschläge [15]
Versteifung in Fehlstellung (z. B. Hammerzehe)	^10/20^ Z	
Versteifung in Neutralstellung	^6/20^ Z	

### Zusätzliche Störungen

#### Schonungszeichen

Da Schonungszeichen einen funktionellen Befund darstellen, der sich durch Gewöhnung und Training bessern kann, sollten sie zum Abschluss des 3. Jahres bemessen werden (Tab. 23).

**Tab. 23:** Aufschlag für Schonungszeichen [12]

Störung	Invalidität	Kommentar zur aktuellen Diskussion
*Muskelminus schonungsbedingt*		Muskelminus belegt eine stärkere Gebrauchsminderung, soll daher in die Bemessung einfließen [13]
Mehr als 2 cm an der *oberen* Extremität	1/20 bis 2/20 A/H/B/F – Wert zusätzlich	
Mehr als 3 cm an der *unteren* Extremität		

#### Längen- und Achsabweichungen

Eine Beinverkürzung ist selten als alleinige Unfallfolge zu verzeichnen, sodass auch hierfür vorgesehene Bemessungen in der Regel nur subsumierend der Basisbemessung hinzuzufügen sind. Meist stehen andere Unfallfolgen im Vordergrund, die maßgeblich sind für die Invaliditätsbemessung (Tab. 24 und 25)!

**Tab. 24:** Aufschlag für Längenabweichungen [12]

Störung	Invalidität	Kommentar zur aktuellen Diskussion
*Beinverkürzung*		Die stärkere Differenzierung erlaubt eine adäquate Bemessung der Gebrauchsbeeinträchtigung gegenüber den Vorschlägen von Klemm et al. [15]
Bis 1 cm	Normvarianz, *keine Gebrauchsbeeinträchtigung*	
Bis 2 cm	^1^/_20_ B	
Bis 3 cm	^2/20^ B	
Bis 4 cm	^3/20^ B	
Bis 5 cm	^5/20^ B	
Mehr als 5 cm	^7/20^ B

**Tab. 25:** Aufschlag für Achsabweichungen [12]

Störung	Invalidität	Kommentar zur aktuellen Diskussion
*Achsabweichungen der Beine*		Die Gebrauchsbeeinträchtigung nimmt mit zunehmender Achsabweichung exponentiell zu, soll daher nicht linear [15] bemessen werden
> 5–10°	^1^/_20_ B	
> 10–15°	^3/20^ B	
> 15–20°	^6/20^ B	
> 20°	^10/20^ B	

#### Arthroseaufschlag

Die Ausprägung der Arthrose nimmt über Jahre zu, die zuzuordnenden Funktionsstörungen ebenso, damit auch die Gebrauchsbeeinträchtigung und soll damit auch – im Gegensatz zu Klemm et al. [13] bemessen werden. Je nach Ausprägung der Arthrose zum Bemessungszeitpunkt zusätzlich bei Kellgren [26] II^0^ 1/20, Kellgren III–IV^0^ 2/20. Diese Bemessung sollte zum Zeitpunkt des 3. Jahres überprüft werden.

Durch Subsumtion des Arthroseaufschlags zur bemessenen Invalidität darf der Wert bei maximaler Funktionsstörung des Gelenks nicht überschritten werden.

#### Thrombosefolgen

Eine zumindest mittelschwere oder hochgradige chronisch-venöse Insuffizienz sollte eine Invaliditätsbemessung durch einen angiologischen Gutachter erfahren, möglichst erst am Ende des 3. Unfalljahres.

Sofern es sich um isolierte Unfallfolgen handeln sollte, gibt die nachfolgende Tabelle Anhaltspunkte über die Größenordnung der jeweiligen Invaliditätsbemessung nach der Gliedertaxe. Bestehen anderweitige, häufig dann auch wesentlichere Unfallfolgen mit Funktionsstörungen, ist die Bemessung nach dem hierfür zur Verfügung stehenden Bemessungsvorschlägen vorzunehmen, die Thrombosefolgen sind dann in subsumierender Weise mit zu berücksichtigen.

Die Bemessung erfolgt nur anhand der Weichteilsituation (Tab. 26).

**Tab. 26:** Aufschlag für Thrombosefolgen [12]

Störung	Invalidität	Kommentar zur aktuellen Diskussion
*Mehrumfang am Unterschenkel bis 1* *cm – Messfehlerbreite*	Keine Invalidität	Ein angiologisches Gutachten kann zu empfehlen sein [15]
*Mehrumfang bis 2* *cm*	^2^/_20_ B	
Mehrumfang mehr als 2 cm mit Pigmentablagerung, Kompressionsstrumpf erforderlich	^4/20^ B	
+ Schwere trophische Störungen	^6/20^ B	
+ Rezidivierendes Ulcus cruris	^8/20^ B	
+ Chronisches Ulcus cruris, nicht mehr therapiefähig	^10/20^ B	

### Gliedertaxenwerte bei Nervenschäden

Zur Gebrauchsminderung durch Nervenschäden wurden keine Diskussionsbeiträge publiziert (Tab. 27 und 28).

**Tab. 27:** Invalidität durch kompletten Verlust einer Nervenfunktion am Arm [11]

Funktionsstörung	Leitsymptome/Hinweise	Invalidität
Vollständige Armplexuslähmung (Lähmung des gesamten Armnervengeflechts)	s. obere und untere Armplexuslähmung	^20^/_20_ A
Obere Armplexuslähmung	Herabhängender, schlaffer Arm in Addition und Innenrotation, Pronationshaltung der Hand	^10^/_20_ A
Untere Armplexuslähmung	Parese der kleinen Handmuskeln und Beuger im Handgelenk (Pfötchenstellung)	^12/20^ A
**Lähmung des**		
*N. radialis (Speichennerv)*		
R. profundus	Parese der Fingerstrecker (Fallhand) und eines Handstreckers	^6/20^ H
Oberarm nach Abgang der Äste zum M. triceps brachii	Zusätzlich auch Parese des anderen Handstreckers und der Armbeugung in Pronationsstellung	^6/20^ A
Kompletter Nerv	Zusätzlich Parese der Armstreckung	^6/20^ A
*N. ulnaris (Ellennerv)*	Parese der Daumenadduktion, (Krallenhand)	^4/20^ A
Handgelenk	Parese der Kleinfingerabduktion, der Daumenadduktion und der anderen Interosseusmuskeln, Krallenhand, Sensibilitätsstörungen D IV/V	^6/20^ H
Kompletter Nerv	Zusätzlich Parese der Flexion der ulnaren Finger und eines Handbeugers	^8/20^ H
*N. medianus (Mittelnerv)*		
Handgelenk	Sensibilitätsverlust D I–III, Parese der Daumenopposition	^6/20^ H
N. interosseus anterior (rein motorisch)	Parese der Flexion der Endglieder von Daumen und Zeigefinger	^4/20^ H
Kompletter Nerv	Zusätzlich Parese eines Handbeugers sowie der langen ulnaren Fingerbeuger	^14/20^ H
*N. radialis und ulnaris*	Kombination der Einzelausfälle	^12/20^ A
*N. radialis und medianus*	Kombination der Einzelausfälle	^16/20^ A
*N. thoracicus longus*	Parese der Abduktion, Anteversion und Außenrotation im Schultergelenk, „Scapula alata“, Instabilität der Schulter	^4/20^ A
N. accessorius (XI. Hirnnerv)	Parese der Abduktion, Anteversion und Außenrotation im Schultergelenk	^4/20^ A
*N. axillaris (Achselnerv)*	Parese der Abduktion, Anteversion und Außenrotation im Schultergelenk, Instabilität der Schulter	^6/20^ A
*N. musculocutaneus*	Parese der Armbeugung in Supinationshaltung	^6/20^ A
*N. suprascapularis*	Eingeschränkte Ad‑, Abduktion und Außenrotation sowie erhöhte Rotatorenmanschetteninstabilität	^2/20^ A

**Tab. 28:** Invalidität durch kompletten Verlust einer Nervenfunktion am Bein [11]

Funktionsstörung	Leitsymptome/Hinweise	Invalidität
Totale Beinplexuslähmung (Plexus lumbosacralis)	Komplette Parese: Hüftbeugung, -streckung, Kniebeugung, -streckung und aller Unterschenkel‑/Fußmuskeln	^20/20^ B
Plexus lumbalis	Parese der Hüftbeugung und -adduktion sowie Kniestreckung	^12/20^ B
Plexus sacralis	Parese der Hüftstreckung und -abduktion, der Kniebeuger und aller Unterschenkel‑/Fußmuskeln	^16/20^ B
**Lähmung des gesamten**		
*N. obturatorius*	Parese der Oberschenkeladduktion	^2/20^ B
*N. ischiadicus (Hüftnerv)*	Parese ischiokrurale Muskulatur, peripher Fußsenker- und Fußheberparese	^16/20^ B
*N. femoralis (Schenkelnerv)*	Parese der Kniestreckung, Sensibilitätsstörung an der Vorderseite des Oberschenkels und Innenseite des Unterschenkels	^10/20^ B
*N. gluteus inferior (Gesäßnerv)*	Parese der Hüftstreckung	^5/20^ B
*N. gluteus superior (Gesäßnerv)*	Parese der Oberschenkelabduktion	^5/20^ B
*N. cutaneus femoris lateralis*	Hier ist lediglich der Schmerz zu bewerten, nicht jedoch die Sensibilitätsstörung	^10/20^ B
*N. peroneus superficialis (oberflächlicher Wadenbeinnerv)*	Parese der Hebung des Fußaußenrandes, Sensibilitätsausfall am Fußrücken	^4/20^ F
*N. peroneus profundus (tiefer Wadenbeinnerv)*	Parese der Fuß- und Zehenhebung	^10/20^ F
*N. peroneus communis (gemeinsamer Wadenbeinnerv)*	Ausfälle von superficialis und profundus	^10/20^ F
*N. tibialis (Schienbeinnerv) Höhe Sprunggelenk*	Parese der Muskulatur der Fußsohle, Sensibilitätsausfall Fußsohle	^8/20^ F
*N. tibialis (Schienbeinnerv) gesamter Nerv*	Zusätzlich Parese der Fuß- und Zehensenkung	^12/20^ F
*N. ischiadicus distal (Ausfall Nn. peroneus communis und tibialis)*	Wie N. peroneus und N. tibialis, zusätzlich Parese der Kniebeugung	^12/20^ B

Läsionen des N. pudendus sind nicht nach der Gliedertaxe zu bewerten

### Invaliditätsbemessung außerhalb der Gliedertaxe

#### Wirbelsäule

Es wird Bezug genommen auf die segmentbezogene Funktionsstörung.

Gemeinsam mit einer eventuellen zusätzlichen Berücksichtigung und Bemessung eines Segmentschadens (s. oben) können im orthopädisch-unfallchirurgischen Bereich maximal 30 % erreicht werden. Nur bei sehr ungewöhnlichen Ausheilungssituationen können allein im orthopädisch-chirurgischen Bereich 30 % überschritten werden. Ansonsten ist dies nur möglich bei zusätzlichen neurologischen Funktionsstörungen, die grundsätzlich in ihrer Bemessung einem nervenärztlichen Sachverständigen überlassen bleiben müssen und – im Falle einer kompletten Querschnittlähmung – bis zu 100 % betragen können.

Beim Ausmessen der statischen Verhältnisse a. p. sowie seitlich eignet sich die Berücksichtigung des bisegmentalen Grund-Deckplatten-Winkels [16].

Fehlstatik durch Achsenknick und Versteifungen der Brustwirbelsäule (bis zum thorakolumbalen Übergang) wirken sich geringer aus.

Die Bemessung für Dornfortsatz- und Querfortsatzfrakturen wurde gestrichen, da funktionell keine Auswirkungen festzustellen sind (Tab. 29).

**Tab. 29:** Invalidität durch Funktionsstörungen und Formstörungen der Wirbelsäule [12]

Funktionsstörung	Invalidität (%)	Kommentar zur aktuellen Diskussion
Stabil verheilter Wirbelkörperbruch Keine oder nur geringe Fehlstatik, bisegmentaler Kyphosewinkel < 10° ohne Störung des sagittalen Profils Ggf. Höhenminderung der angrenzenden Bandscheibe ohne wesentliche segmentbezogene Funktionsstörung	5	Keine sonstigen Vorschläge
Stabil verheilter Wirbelkörperbruch Leichter Achsenknick, bisegmentaler Kyphosewinkel 10° bis < 20°, sagittales Profil noch erhalten Ggf. Höhenminderung der angrenzenden Bandscheibe mit mäßiger segmentbezogener Funktionsstörung	10	
*Stabil* verheilter Wirbelkörperbruch Statisch wirksamer Achsenknick bisegmentaler Kyphosewinkel > 20°, sagittales Profil gestört (Lotlinie C7/S1 mehr als 50 mm vor hinterem Anteil der Endplatte S1) oder Verheilter Wirbelkörperbruch mit verbliebener segmentaler Instabilität	20	
Versteifung bis zu drei Segmenten der LWS (einschließlich thorakolumbaler Übergang) oder der HWS (unterhalb HWK 2)	20	
Verheilter Wirbelkörperbruch mit erheblicher Störung des sagittalen Profils (Lotlinie C7/S1 mehr als 70 mm vor hinterem Anteil der Endplatte S1), (bisegmentaler Grund-Deckplatten-Winkel > 30°) und radiologisch objektivierbarer segmentaler Instabilität	30	
Operative Versteifung von drei und mehr Bewegungssegmenten der HWS (unterhalb HWK 2), der LWS und des thorakolumbalen Übergangs	30	

*HWK* Halswirbelkörper, *HWS* Halswirbelsäule, *LWS* Lendenwirbelsäule

#### Becken [10]

Funktionsstörungen des Urogenitalapparats müssen urologischerseits objektiviert und – außerhalb der Gliedertaxe – bemessen werden, nach AUB 88 mit additivem Zusammenführen der Bemessungen auf beiden Fachgebieten. Sofern die AUB 99 und folgende zur Anwendung kommt, ist eine subsumierende Gesamtbemessung vorzunehmen, ggf. dann auch unter Mitberücksichtigung eventuell verbliebener neurologischer Funktionsstörungen, die nervenärztlicherseits zu objektivieren und zu bemessen sind.

Sofern Nervenfunktionsstörungen die Funktion des Beines beeinträchtigen, sind diese gesondert nach der Gliedertaxe – nervenärztlich – zu bemessen (Tab. 30).

**Tab. 30:** Invalidität durch Funktionsstörungen des Beckens [12]

Funktionsstörung	Invalidität (%)	Kommentar zur aktuellen Diskussion
Vordere Beckenringfraktur (ein- oder beidseitig) mit geringgradiger Beeinträchtigung der Steh- und Gehfähigkeit	5	Ähnlichkeiten der Staffelung der Funktionsstörungen als Grundlage der Bemessung sind erkennbar [16], wird hier durch das Kriterium der hochgradigen Beeinträchtigung der Steh- und Gehfähigkeit ergänzt
Beckeninstabilität oder Formstörung mit geringgradiger Beeinträchtigung der Steh- und Gehfähigkeit	10	
Beckeninstabilität oder Formstörung mit mittelgradiger Beeinträchtigung der Steh- und Gehfähigkeit	20	
Beckeninstabilität oder Formstörung mit hochgradiger Beeinträchtigung der Steh- und Gehfähigkeit	30	

Azetabulumfrakturen werden funktionell dem Hüftgelenk zugerechnet

#### Thorax

Fehlverheilte Rippenfrakturen können restriktive Atemstörungen hinterlassen, die durch den hierfür kompetenten Gutachter zu objektivieren und zu bemessen sind. Eine Interkostalneuralgie bedarf einer neurologischen Abklärung. Die Bemessungen auf mehreren Fachgebieten sind nach AUB 88 additiv, nach AUB 99 subsumierend zusammenzuführen (Tab. 31).

**Tab. 31:** Invalidität durch Funktionsstörungen des Thorax [12]

Funktionsstörung	Invalidität (%)	Kommentar zur aktuellen Diskussion
Brustbeinpseudarthrose	5	Übereinstimmung mit Klemm et al. [16]
Fehlverheilte Rippenfraktur(-en) mit Beeinträchtigung der Atemmechanik	10	

#### Bauchdecken

Unfallfolgen an den Bauchorganen (Milzverlust und Teilverlust des Darmes etc.) sind zu objektivieren und zu bemessen (Tab. 32).

**Tab. 32:** Invalidität durch Bauchdecken – Narben, Hernien [12]

Funktionsstörung	Invalidität (%)	Kommentar zur aktuellen Diskussion
Narbige Umwandlungen eines Teiles der Bauchwandmuskulatur	5	Weitgehende Übereinstimmung mit Klemm et al. [16]
Kleine Bauchwandhernie (bis Tischtennisballgröße)	10	
Bauchwandhernie (bis Faustgröße)	15	
Größerer Bauchwandbruch	20	
„Landkarten-Bauchdecke“ mit grober muskulärer Insuffizienz	25	

### Fazit

Diese Tabellen sollen Inkonsistenzen der bisherigen Bemessungsempfehlungen verschiedener Autoren vermeiden.

Gegenüber den Tabellenvorschlägen von 2022 wurden nach eingehender Diskussion der aktuellen Bemessungsempfehlungen manche Revisionen vorgenommen. In den Kommentaren zu den einzelnen Verletzungsfolgen werden Hinweise und Begründungen für Änderungen ausgeführt. Die Bemessungen wurden umgestellt auf Zwanzigstel der Gliedmaßenwerte. Der Diskurs verschiedener Autoren hält Tabellenempfehlungen in einem dynamischen Prozess, der begründete Änderungsvorschläge aufnimmt.

Dieser Tabellen führen somit die bisher nebeneinanderstehenden Tabellen zu einheitlichen Bemessungsempfehlungen muskuloskelettaler Verletzungsfolgen zusammen. Wie bei allen Tabellenwerken muss sich der materielle Wert ihrer Empfehlungen in der täglichen Anwendung bewähren.

## Abkürzungen

A: Armwert
AUB: Allgemeine Unfallversicherungsbedingungen
B: Beinwert
CRPS: complex regional pain syndrome
D: Daumenwert
DGOU: Deutsche Gesellschaft für Orthopädie und Unfallchirurgie
DKOU: Deutscher Kongress für Orthopädie und Unfallchirurgie
F: Fußwert
Fi: Fingerwert
GUV: Gesetzliche Unfallversicherung
H: Handwert
HWK: Halswirbelkörper
HWS: Halswirbelsäule
LWS: Lendenwirbelsäule
MdE: Minderung der Erwerbsfähigkeit
N: Nervus
PUV: Private Unfallversicherung
VSOU: Vereinigung Süddeutscher Orthopäden und Unfallchirurgen
